# Frailty's Prevalence and the Association with Aging-Related Health Conditions in Chinese Community Dwelling Elderly

**DOI:** 10.1155/2022/1748162

**Published:** 2022-08-16

**Authors:** Hongxiao Lin, Dongyan Wang, Shanjun Ma, Yan Suo, Peng Zhou, Qing Zhao, Juan Liu, Guoxian Ding

**Affiliations:** ^1^Department of Geratology, The First Affiliated Hospital of Nanjing Medical University, 300 Guangzhou Road, Nanjing 210029, China; ^2^Department of Osteoporosis, The First Affiliated Hospital of Kangda College of Nanjing Medical University, 6 Zhenhua East Road, Lianyungang 222000, China; ^3^Department of Osteoporosis, The Affiliated Lianyungang Hospital of Xuzhou Medical University, 6 Zhenhua East Road, Lianyungang 222000, China; ^4^Department of Geratology, Xinpu Community Health Service Center, 146 Nanji North Road, Lianyungang 222000, China

## Abstract

In this paper, we have investigated the frailty's prevalence and the association with aging-related health conditions in Chinese community dwelling elderly aged ≥60 years in Lianyungang City of China. In this regard, participants were 1,072 adults aged ≥60 years from Houhe Community of Lianyungang City of China. All the enrolled participants were tested for following parameters: (1) the related risk factors of frailty: including economic status, personal health, understanding and communication skills, and mental and psychological status; (2) aging-related health conditions related to frailty: Charlson's comorbidity index (CCI), Mini Nutritional Assessment Short Form (MNA-SF), Patient Health Questionnaire-9 (PHQ-9), and Generalized Anxiety Disorder 7-item (GAD-7); (3) body composition, physical strength, and function testing: appendicular skeletal muscle mass index (ASMI), grip strength, five-repetition sit-to-stand test, 6 m walking speed, and strength assistance rise-climb-fall (SARC-F); (4) assessment of the degree and severity of frailty: physical frailty phenotype (PFP), Morse fall scale (MFS), and activities of daily living (ADL). The frailty's prevalence among the elderly aged ≥60 years in the community of Lianyungang City was 13.8%, 55.4% were prefrail, and 30.8% were robust. The independent risk factors of frailty were age, appendicular skeletal muscle mass index, sarcopenia, education, nutrition, and strength assistance rise-climb-fall (*P* < 0.05). Aging-related health conditions were associated with frailty, including sarcopenia, nutrition, and falls. However, mental and psychological statuses were not significantly associated with frailty.

## 1. Introduction

Frailty is a physiological syndrome indicating low overall reserve capacity of the body due to the decline of multiple systems, which causes clinical manifestations and adverse outcomes [1–5]. Compared with nonfrail elderly, the risk of death of frail elderly increased 15–50% [6]. According to a research conducted in the USA, the average yearly medical costs of frail old persons were three times higher than those of nonfrail senior people. In these studies, numerous factors have been identified which are very important as far as this ratio in elder patients is concerned [7].

China, formally known as the People's Republic of China, is a nation in East Asia. It is the world's most populous country, with a population of nearly 1.4 billion people. China shares borders with 14 countries and spans five time zones, the second most of any country in the world behind Russia. The population aging in China increases rapidly. In 2020, China's population of people aged 60 and more will number 264 million, accounting for 18.7% of the population's total. In 2050, the number is expected to reach 483 million, accounting for more than 30% of the entire population. The older population is enormous, and their health is complicated; they are also the most susceptible group in terms of health [8–10]. Because the concept of frailty can well assess health status of the elderly and predict the prognosis of the elderly [11], it has become a focus in modern geriatric research [12, 13]. Geriatric research also includes advances in the diagnosis, treatment, and pathophysiological disorders related to aging, such as arthritis, renal impairment, urine incontinence, cognitive impairments, chronic joint and bone pain, neurological illnesses, and vision and hearing impairment. Additionally, it is very important that these problems are required to solve on priority bases and thus various scientists have recommended techniques as described above; however, specialized approaches are needed to be developed.

In this manuscript, we have extensively used one of the most widely and well-known validation approaches, i.e., physical frailty phenotype (PFP) scale, which is used to examine the frailty's prevalence and the respective association with aging-related health conditions in Chinese community dwelling elderly. Likewise, this approach is verified by conducting experimental studies, where number of patients participated in each experiment is described in the subsequent section.

The rest of the article is arranged as follows.

In section labeled as Methods, the proposed technique along with how and why various patients are encouraged to be part of this study is reported. Moreover, a detailed selection and rejection criterion is defined for both groups. More importantly in Section 3, a detailed discussion is provided on the underlined data collected and which mechanisms are used for it. In Section 4, results of the scheme under consideration are verified through experimental setup and presented in both textual and graphical formats. A discussion section on the overall scenario, i.e., from problem statement to the conclusive remarks, is reported in Section 5, whereas summary is presented in the last section.

## 2. Methods

### 2.1. Participants

A total of 1,072 elderly people aged ≥60 years in Houhe Community of Lianyungang City were screened from August 2020 to July 2021. To choose a representative community cohort of people aged 60 and up, a multistage cluster random selection procedure was utilized. Participants in this study completed a questionnaire as well as clinical examinations. All participants signed a written informed consent form.

## 3. Data Collection

Collection of data is the process of gathering and analyzing organized data on certain variables in order to answer important questions and measure outcomes. Data collection is a crucial phase of every research domain and process in approximately every field of academia such as social and physical, business, and humanities. We will go through each of them individually in this part.

### 3.1. General Demographic Data and the Related Risk Factors of Frailty

Demographic data were gathered from the members, including age, sex, status of the marital, residential location (current), education, occupation, personal health, economic status, understanding and communication skills, and mental and psychological status.

### 3.2. Assessment of Aging-Related Health Conditions Related to Frailty

All the enrolled participants were screened and tested for the following tests: CCI, MNA-SF, PHQ-9, and GAD-7. CCI is a way of identifying patient comorbidities using the ICD diagnostic codes obtained in data related to administrative process like hospital abstracts. Every category of comorbidity is assigned a weight (from 1 to 6) depending on the attuned risk of mortality or resource utilization, and a weighted sum of all possible results in a single comorbidity score for a patient. With a score of 0, there were no comorbidities found.

### 3.3. Assessment of Body Composition, Physical Strength, and Function Testing

Muscle mass was measured using bioimpedance analysis (BCA-2A, THTF, China). The AWGS 2019 defined the cutoffs for height-adjusted muscle mass (ASM/height2, ASMI): less than seven kg/m^2^ in men and less than five point seven kg/m^2^ in women. AWGS 2019 consensus defined the diagnostic criteria: handgrip strength less than twenty-eight kg for men and less than eighteen kg for women was considered “low muscle strength”; 6 m walk less than 1.0 m/s and five-repetition sit-to-stand test greater than or equal to 12 seconds were deemed low physical performance.

SARC-F (rise-climb-fall) strengthening support consists mostly of five items: (i) have you walked 400 meters in a row so far this week? How many times have you walked like this before? (ii) Could you tell me how difficult it is to cross a room? (iii) Is getting out of bed or a chair difficult? (iv) How difficult are the 10 steps? (v) How many times have you fallen in the previous year? “Positive” was assigned to those who satisfied four of the requirements.

### 3.4. Assessment of the Severity of Frailty

The severity of frailty was assessed by Fried's physical frailty phenotype (PFP) scale that is based on five different criteria such as exhaustion, slowness, weakness, shrinking, and physical inactivity. Participants who met none of the requirements were labeled “robust,” whereas those who met 1–2 criteria were labeled “prefrail,” and those who met three criteria were labeled “frail.”

Morse fall scale (MFS) mainly contained five items: (i) whether there has been a fall in the past three months; (ii) more than one disease; (iii) receive medication; (iv) gait/movement; and (v) mental state. Those meeting ≥4 criteria were considered “positive.”

Physical activity was measured using the activities of daily living (ADL) scales, which included (i) the Basic Activities of Daily Living Ability Scale (BADL): covering 6 items such as going to the toilet, eating, putting on clothes, grooming (tidy, hair, nails, hands, face, clothing), getting out of bed, and taking a bath; and (ii) the Instrumental Activities of Daily Living Ability Scale (IADL): covering 8 items such as going out, shopping, and taking. The individuals were divided into four categories: severe, moderate, mild, and strong.

### 3.5. Statistical Analyses

Measurements related to the collected data were represented in the form of mean ± and standard deviation, variance's analysis was used for the assessment among groups, data's enumeration was expressed as frequency or percentage (%), and chi-square test is used for matching or similarity computation between groups. Binary logistic stepwise regression analysis was performed, the degree of frailty was based on the prefrail (0 = robust, 1 = prefrail) and frail (0 = prefrail, 1 = frail) as the dependent variables. All tests were two-tailed, and *P* < 0.05 was measured statistically noteworthy.

## 4. Results

This section, namely, “Results” is described to be the section where we need to provide the proposed study's conclusions depending on the technique used to collect data. The collected or observed results are described below one by one.

### 4.1. Frailty's Prevalence and Demographic Characteristics

The frailty's prevalence among the elderly aged ≥60 years in the community of Lianyungang City was 13.8%, 55.4% were prefrail, and 30.8% were robust. The following were the effects of demographic variables on the frailty of the elderly in the community. Frailty was found to be more prevalent in males than in women, with 11.5 percent of men and 15.8 percent of women being frail, respectively. Frailty was more common in women than in men among the elderly. Frailty became more prevalent as people became older. Frailty was found in just 2.1 percent of individuals aged 60 to 69 years, whereas 23 percent of those aged 80 years were considered feeble. In addition, people who were widowed had a lower level of education, had no work, and had a greater frequency of frailty, as shown in Table 1.

### 4.2. The Correlation of Aging-Related Health Conditions with Frailty

Single-factor analysis showed that the risk factors of frailty were sex, age, marital status, education level, occupation, urinary incontinence, CCI, the number of oral medications, nutrition, ADL, and falls (*P* < 0.05, as shown in Table 2).

### 4.3. The Correlation of Sarcopenia and Body Composition with Frailty

The prevalence of sarcopenia was 11.2% among the overall enrolled subjects and was 11.7% in male elderly and 10.8% in female elderly. The prevalence of suspicious sarcopenia was 43.6%. Single-factor analysis showed that sarcopenia, BMI, and ASMI were the risk factors of frailty (*P* < 0.05, as shown in Table 3).

### 4.4. Logistic Regression Analysis of the Influencing Factors of Frailty

The prefrail (0 = robust, 1 = prefrail) (Table 4) and the frail (0 = prefrail, 1 = frail) (Table 5) were selected as the dependent variable, respectively, and the factors with statistical differences in univariate enquiry were used as self-determining variables for binary logistic regression analysis. The outcomes exposed that the independent risk factors of prefrailty were sex, occupation, sarcopenia, ASMI, residence, drinking, CCI, and SARC-F (*P* < 0.05); the independent risk factors of frailty were age, ASMI, sarcopenia, education, nutrition, and SARC-F (*P* < 0.05, Tables 4 and 5).

## 5. Discussion

In this study, we found that the frailty's prevalence among the elderly aged ≥60 years in the community of Lianyungang City was 13.8%, and 55.4% of them were prefrail. Nguyen et al. [14] reported that the frailty's prevalence among the elderly in the Chinese community was 5–31%, and the overall frailty's prevalence among the elderly 65 years and older was about 10%. CHARLS showed that the frailty's prevalence among the elderly in the community was 7.0% [15]. These results indicated that the frailty status of the elderly in Lianyungang community was serious. This study and other studies suggest that the elderly in the community of prefrailty account for a larger proportion of the elderly [16, 17]. At present, many studies in China focus on the occurrence and prevention of frailty, but frailty is a short and reversible process [18–20]. The risk of developing into frailty at 18 months for the elderly in the prefrailty stage is about 5 times that of the elderly without frailty, and frailty can be transferred to prefrailty [21].

In addition, the disparities in frailty incidence among different groups of subjects in our study were consistent with other studies in China [22, 23]. We found that frailty prevalence differed by sex, since women had a significantly higher frailty's prevalence in the elderly, consistent with Zheng's study [24]. With advancing age, widowed marital status, and lower education level, the frailty's prevalence increased. These findings were consistent with a large, nationally representative sample study that examined the incidence of frailty among Chinese older adults aged 60 years or older [15]. However, mental and psychological statuses were found to be not significantly associated with frailty in our study, different from previous results [25].

More than 65 percent of old and frail persons had several chronic conditions, according to Chen et al. [26], with 55 percent having trouble eating and over 50 percent having mobility issues. Proton pump inhibitors, diuretics, hypoglycemic medicines, and antihypertensive medications are only a few of the therapies that might make you fragile [27]. Frail persons using ten or more medicines were six times more likely to die, according to Herr et al. [28]. As a result, in the treatment of chronic illnesses in the elderly, the benefits and drawbacks of pharmaceutical therapies should be weighed.

Fried et al. proposed the “frailty cycle model” and believed that the core of frailty is sarcopenia, which plays an important role in the occurrence and development of frailty. The results of this study showed that sarcopenia was closely related to frailty of the elderly in the community and was an independent risk factor for frailty and prefrailty. Other studies have shown that low body weight and low BMI were positively correlated with increased prevalence and morbidity of sarcopenia [29], and pace could independently predict disability, cognitive dysfunction, falls, and death [30].

Our study has several strengths. First, most studies on frailty in China focus on hospitalized patients, but there are still few studies on frailty among the community. This study can be used as a reference for the frailty's prevalence among urban residents in eastern China. Second, our study conducted a comprehensive screening and evaluation of the frailty's prevalence and the association with aging-related health conditions in Chinese community dwelling elderly. Third, our study enrolled relatively large sample of typical elderly residents living in the community. Our study has several limitations. First, we used a large number of questionnaires in this study; therefore, self-report bias and recall bias are inevitable. Second, we may have underestimated the prevalence of depressive symptoms, which may affect the results. Third, our study is a cross-sectional study, and our results should be confirmed by longitudinal studies.

## 6. Conclusion

In this study, we have observed that frailty status of the elderly in Lianyungang community was serious. We found that the aging-related health conditions were significantly associated with frailty. It is very important to formulate targeted intervention measures to delay or even reverse the frailty. Frailty was prevalent among the elderly aged 60 years in the Lianyungang City community, with 13.8 percent frail, 55.4 percent prefrail, and 30.8 percent robust. Age, appendicular skeletal muscle mass index, sarcopenia, education, diet, and strength assistance rise-climb-fall were all independent risk variables for frailty (P0.05). Frailty has been linked to aging-related health issues such as sarcopenia, nutrition, and falls. However, mental health and psychological well-being were not shown to be substantially linked to frailty.

## Figures and Tables

**Table 1:** The influence of demographic characteristics on frailty in the elderly in the community (*n* = 1,072).

Variables	Stratification	Degree of frailty			^*2*^	*P*
		Robust	Prefrail	Frail		
Sex					11.158	0.004
	Male	135	297	56		
	Female	195	297	92		

Age (years)					140.387	<0.001
	60∼69	220	103	7		
	70∼79	297	273	24		
	≥80	32	82	34		

Marital status					13.999	0.001
	Married	305	540	121		
	Unmarried	1	1	0		
	Divorce	2	4	1		
	Widowed	22	48	26		
	Others	0	1	0		

Education					9.589	0.008
	Illiterate	33	68	36		
	Elementary	51	112	40		
	Middle	146	238	46		
	High	81	46	18		
	College	19	18	8		

Residence Status					3.162	0.206
	Solitude	20	60	45		
	With spouse	265	459	75		
	With family	45	103	27		

Occupation					6.040	0.049
	Civil servant	4	5	2		
	Teacher	2	9	2		
	Soldier	1	2	0		
	Institution staff	37	56	17		
	Enterprise staff	242	424	94		
	Farmer	14	29	10		
	Business	3	15	2		
	No occupation	27	54	21		

**Table 2:** The influence of aging-related health conditions on the frailty in community dwelling older people (*n* = 1,072).

Variables	Stratification	Degree of frailty			*χ* ^2^	*P*
		Robust	Prefrail	Frail		
Smoking					2.357	0.308
	No	250	435	117		
	Yes	48	117	22		
	Quit	32	22	9		

Drinking					4.359	0.113
	No	235	449	118		
	Yes	85	129	25		
	Quit	10	16	5		

Pain					2.867	0.239
	No	216	419	100		
	Yes	111	168	42		

Urinary incontinence					21.359	<0.001
	No	304	545	118		
	Mild	5	2	1		
	Moderate	20	41	20		
	Severe	1	6	9		

Sleeping					2.545	0.280
	No	257	476	110		
	Yes	73	118	38		

CCI					13.251	0.001
	Low	148	178	20		
	Moderate	179	408	120		
	High	3	8	7		
	Very high	0	0	1		

Types of oral drugs					15.410	0.004
	0	246	373	97		
	1∼4	81	208	46		
	≥5	3	13	5		

MNA-SF					19.230	0.001
	Normal	0	1	2		
	Nutritional risk	15	50	20		
	Malnutrition	315	543	126		

MMSE					17.752	<0.001
	Normal	179	310	51		
	Nutritional risk	119	239	63		
	Malnutrition	32	45	34		

PHQ-9					3.938	0.140
	No	319	567	137		
	Mild	9	21	8		
	Moderate	2	4	1		
	Moderately severe	0	1	2		
	Severe	0	1	0		

GAD-7					5.369	0.0658
	No	308	564	133		
	Mild	16	19	8		
	Moderate	3	7	3		
	Moderately severe	1	3	3		
	Severe	2	1	1		

ADL					10.474	0.005
	No	254	468	98		
	Mild	71	109	35		
	Moderate	5	17	12		
	Severe	0	0	3		

MFS					34.364	<0.001
	No	307	501	108		
	Yes	23	93	40		

**Table 3:** The influence of sarcopenia and body composition status on frailty in the community dwelling older people (*n* = 1,072).

Variables	Stratification	Degree of frailty			*χ* ^2^/F	*P*
		Robust	Prefrail	Frail		
Sarcopenia					445.894	<0.001
	No	275	207	3		
	Probable	55	297	115		
	Confirmed	0	81	4		
	Severe	0	9	26		

SARC-F					34.364	<0.001
	No	307	501	108		
	Yes	23	93	40		

BMI					16.201	0.013
	Thin	12	32	10		
	Normal	103	246	51		
	Overweight	152	219	54		
	Obesity	63	97	33		

ASMI		7.60 ± 1.42	7.23 ± 1.52	7.19 ± 1.52	7.466	0.001

SARC-F; BMI; ASMI.

**Table 4:** Logical regression analysis of risk factors for the elderly in the community.

Variables	*β*	SE	Wald	OR	95% CI	*P*
Sex	−1.215	0.221	30.186	0.297	0.192–0.458	<0.001
Occupation	0.186	0.074	6.361	1.204	1.042–1.391	0.012
Sarcopenia	2.352	0.190	153.797	10.501	7.242–15.228	<0.001
ASMI	−0.320	0.067	22.756	0.726	0.637–0.828	<0.001
Residence	−0.387	0.184	4.435	0.679	0.474–0.974	0.035
Drinking	−0.524	0.193	7.329	0.592	0.406–0.865	0.007
CCI	0.589	0.169	12.159	1.803	1.294–2.511	<0.001
SARC-F	0.619	0.286	4.690	1.858	1.061–3.253	0.030

ASMI; CCI; SARC-F.

**Table 5:** Logical regression analysis of risk factors for the elderly in the community.

Variables	*β*	SE	Wald	OR	95% CI	*P*
Age	1.109	0.177	39.142	3.032	2.142–4.293	<0.001
ASMI	0.185	0.091	40126	1.203	1.007–1.438	0.042
Sarcopenia	1.199	0.182	43.444	3.316	2.322–4.737	<0.001
Education	−0.314	0.106	8.711	0.731	0.593–0.900	0.003
MNA-SF	−0.775	0.327	5.616	0.461	0.243–0.875	0.018
SARC-F	0.661	0.261	6.412	1.936	1.161–3.228	0.011

ASMI; MNA-SF; SARC-F.

## Data Availability

The data used to support the findings of this study are available from the corresponding author upon request.
